# The Construction Strategy of a New Model of College Students' Psychological Education under the Network Environment

**DOI:** 10.1155/2022/1952840

**Published:** 2022-06-20

**Authors:** Bin Cai

**Affiliations:** School of Computer Science, Minnan Normal University, Zhangzhou, China

## Abstract

Understanding the interests and needs of online health education for college students, exploring the concepts, procedures, models, and approaches of health plans, learning about mental health online, and developing a comprehensive online mental health education plan for as many college students as possible are always very popular. Based on the development and support of online mental health education for students, from the perspectives of teachers and college students, this paper investigates online mental health education for college students in a city, combined with data interviews and Delphi routes; through electronic questionnaires, 900 college students and 30 students were selected by faculty members to conduct an investigation. With descriptive statistics, reliability and availability, chi-square tests, and other options, this paper examines data on student Internet usage and current status and we have the Psychiatry Network. The results show that 91.75% of college students study online every day and 61.72% spend more than 4 hours online every day. Satisfaction with the Internet has a certain impact on the online application and use of the health college education. Students' online motivations and behaviors are multicultural. In order to build a mental health education network, educators believe that the primary goal should be to improve the mental health of college students.

## 1. Introduction

Mental health is the foundation of cognition. Only by having a healthy university environment can students' morality, intelligence, physique, and beauty be improved in all aspects. College students are the backbone of the nation's future, leading to high expectations from individuals and parents [1]. Mental health not only affects the normal education, life, and happiness of college students but also affects the overall quality of Chinese art. It is a major event related to the rise and fall of the country and the survival of the nation. With the advent of the era of knowledge economy and information society, people's pace of life has accelerated significantly, social competition is becoming increasingly fierce, social members are under increasing pressure, and the number of patients with mental diseases is increasing day by day. As a special group with high expectations from society and parents, college students also face greater pressure than other peer groups. The school stage is a period of rapid development in physiology and psychology. It is a transitional period in which individual psychology rapidly moves towards maturity but not yet fully matures [2, 3]. In recent years, the rapid development of computer and network technology has brought many new features to the mental health of college students. College students can share the best resources on the network through the Internet, obtain information more easily, and communicate more easily. However, while the Internet is convenient for students to study and live, it also has many disadvantages for students' health. Many college students do not know how to restrain and control themselves when surfing the Internet. They are addicted to the illusory world of the Internet and cannot free themselves. They suffer from various Internet psychological obstacles such as Internet dependence, Internet loneliness, and Internet addiction syndrome. With the impact and subversion of the Internet tide, the form, content, and integration of student health education have undergone major changes. The psychiatric education standards have difficulty adapting to the major problems brought by the Internet to the psychiatric education in colleges and universities [4]. Therefore, for health educators in colleges and universities, it has become a rapid research topic to strengthen the research of mental disciplines in the network environment and how to better educate students to carry out mental health education in the network environment [5].

## 2. Literature Review

Taghvaei et al. found that as the Internet slowly entered all aspects of public life, it not only had a positive impact on the country and people but also had a negative impact on human psychology [6]. Zhang et al. studied human behavior, mental health, education, and social relations in the network environment, which has become an important part of the research [7]. Zhao et al. believed that mental health research in the network environment not only is a new study of mental health but also plays an important role in supporting the further development of mental illness [8]. Allen et al. found that Western countries, led by the United Kingdom and the United States, were the first to become popular on the Internet. After studying the relationship between the emergence of the Internet environment and human psychological changes, scientists found that the Internet environment can make the elderly change their minds [9]. In the 1970s and 1980s, the “problem-solving-centered” training mode appeared in Britain. Its training work is mainly composed of three parts: preparation before professional training, professional training and on-site work, and advanced professional training. The British Psychological Society stipulates the minimum qualifications for workers: graduate degree or above, teacher qualification certificate, more than two years of teaching experience with children and adolescents, at least two years of educational psychology training after graduate degree, etc. Alégroth and others found that, since the 1980s, France has also set up special training programs, including two parts of trainees' professional learning and internship [10]. Qualification requirements for workers in France were two years of psychology major in university, at least three years of teacher training, and five years of primary school or preschool work experience. The training of school mental health educators in the United States is mainly based on the “scientist practitioner” model, combining research and practice. Applicants should enter the school psychology major taught by the American Association of school psychologists and the American Psychological Society. Marcial and Launer and others found that 20% of people will have “Internet addiction” in the network environment through statistics and analysis of the questionnaire results. They need to surf the Internet every day, and it is difficult to get away from the network environment. In comparison, only 12% of people think that the Internet will bring them a sense of ease and pleasure [11]. Pereira et al. separate the concept of cyber health from that of mental network and study it as a separate concept. However, their concept of cyber health still starts from the concept of mental health and does not understand the importance of the cyber environment [12]. Yasui et al. found that other researchers in cyber psychiatry studies did not account for the merits of disrupting cyber environmental processes [13].

To understand the network and mental health of high school students in a city, this study explores the prevention and improvement of high school students' mental health and college time network and provides a foundation for supporting the development of higher education students' mental illness. According to the development and use of online health services for male and female college students in a city, Yusuwan, New Mexico, found the key points that can improve the mental health of current college students in online learning and gave tips and suggestions to improve the effectiveness of online education for college students' mental health [14]. Based on interest and demand for online health education, more research is required to develop prevention and develop and clean online content and programs for preventive health education, as shown in Figure 1.

## 3. Research Methods

According to the principles of random sampling and convenient sampling, a total of 900 college students were randomly selected from full-time universities, independent colleges, vocational and technical colleges, and colleges in a city. According to the five inclusion criteria of psychology professional background, master's degree or above, full-time mental health education, intermediate professional title or above, and more than 3 years of experience, 30 college mental health educators in a city were randomly selected as the survey objects.

Firstly, we made a statistical description of the distribution and recovery of the questionnaire, the sociodemographic characteristics of the sample, and the use of Internet by college students. Then, EpiData was used to establish the database, Spss17.0 software was used to evaluate the reliability and validity of the questionnaire, and chi square test, analysis of variance, correlation analysis, and multiple stepwise regression analysis were performed on the survey data.

Nine mental health professionals were specially invited to complete interviews with experts on the selection criteria of the questionnaire for “Research on the Construction of College Students' Health Network.” In the first round of preresearch, experts put forward suggestions on adding, modifying, or deleting the questionnaire items based on the preliminary data analysis and research results, as well as the preliminary design of the questionnaire and the author prepared options; in the second part of the interview, the experts removed items with an average score of less than 3 and a difference of more than 40% and continued to apply the average Score 3∼ of expert opinion. The coefficient of variation is 20% to 40%; in the third part of the expert interview, the importance and effectiveness of the measures will be reevaluated, and the weight of the indicators will be consulted. We sorted out the expert consultation questionnaire data, calculated the expert enthusiasm coefficient, expert authority degree coefficient, expert opinion coordination coefficient, and expert opinion variation coefficient using spss170, selected appropriate indicators, and tested the reliability and authority of the consultation results [15].

### 3.1. Selection of Consulting Experts

According to the selection criteria of experts with psychology- and pedagogy-related background and intermediate professional title or above, who engaged in college students' mental health education and research for more than 5 years, a total of 9 experts were invited in this study, most of whom are the (deputy) director of the mental health education and psychological counseling center of a provincial university, and all of them have rich theoretical basis and practical accumulation of college students' mental health education. Among them, four experts have doctoral degrees, four experts have master's degrees, and one expert has bachelor's degrees. The professional background covers psychology, management, pedagogy, medicine, and other disciplines. At the same time, the age range of experts is 36∼66 years, and the average age is 48 years. There are 6 experts who have worked for more than 10 years, of which 3 have worked for more than 20 years. In addition, 2 experts have positive and senior professional titles and 5 experts have deputy senior professional titles. In conclusion, the consulting experts have a high degree of professional authority and familiarity with the contents of this study (see Table 1 for details).

### 3.2. Expert Positive Coefficient

This study takes the recovery rate of consultation questionnaire as the index. The higher the recovery rate of questionnaire, the higher the positive coefficient of experts. In the first presurvey round, 2 paper versions and 7 electronic versions of expert consultation questionnaires were distributed. Experts were invited to score the importance and feasibility of the initial items at five levels, experts' opinions were collected on the index system of the initial questionnaire, and experts' questions were answered in time. After one week, a total of 9 effective expert consultation questionnaires were recovered, and the positive coefficient of experts reached 100%.

The second and third rounds of formal expert consultation sent 9 electronic questionnaires respectively. Each consultation questionnaire includes filling in instructions, importance and feasibility scores, index weights, and judgment basis. The two rounds of formal consultation are one week apart. In the second round of formal consultation, there were two expert questionnaires with individual missing options. The corresponding experts were contacted in time for supplement. Finally, nine effective consultation questionnaires were recovered in the two rounds of formal consultation, and the expert positive coefficient was 100% [16].

### 3.3. Expert Authority Coefficient

The judgment basis (Ca) and familiarity (Cs) are the two determinants of the expert authority coefficient (Cr), and the calculation formula is as follows [17]:

(1) $$\begin{array}{c} \text{Cr}=\frac{\left(Ca+Cs\right)}{2}. \end{array}$$

This study selects four judgment bases, practical experience, theoretical basis, peer understanding, and intuitive judgment and gives three-level quantitative values. At the same time, experts' familiarity is divided into five levels: “very familiar,” “relatively familiar,” “general,” “relatively unfamiliar,” and “unfamiliar,” and different quantitative values are given (see Table 2 for details) [18].

According to the experts' scores on the educators' questionnaire, the first-level index expert authority coefficient is between 0.763 and 0.885, with an average of 0.810. The coefficient of expert authority degree of secondary index ranges from 0.712 to 0.806, with an average of 0.762. According to the scores of experts on the questionnaire of college students, the authority degree coefficient of the first-class index experts is between 0.786 and 0.822, with an average of 0.803. The coefficient of expert authority degree of secondary index ranges from 0.719 to 0.822, with an average of 0.765. In this study, the degree coefficient of expert authority is greater than 0.70, and the average degree coefficient of expert authority at all levels reaches or approaches 0.80, indicating that the degree of authority of experts on the research content is very high.

### 3.4. Coordination Coefficient of Expert Opinions

In this study, Kendall harmony coefficient is selected to judge the consistency of expert opinions. The closer the Kendall harmony coefficient is to 1, the higher the consistency of expert opinions is. Kendall harmony coefficient is in the range of 0.4∼0.5, indicating that the prediction result is desirable, higher than 0.7, which can be considered as a very high degree of expert consistency. In the second round of formal consultation, the Kendall harmony coefficients of the overall index importance and feasibility of the educators' questionnaire were 0.432 and 0.417, respectively, and the Kendall harmony coefficients of the overall index importance and feasibility of the college students' questionnaire were 0.584 and 0.517, respectively, reaching a basically consistent level. In the third round of formal consultation, the Kendall harmony coefficient of the two types of questionnaire indicators increased significantly, which shows that the expert opinions tend to be consistent. The Kendall harmony coefficient of the overall index importance and feasibility of the questionnaire reached 0.7, and the *p* value was less than 0.05, indicating that the expert evaluation results are desirable (see Tables 3to 4 for details).

#### 3.4.1. Index System Screening Results

In the first preliminary evaluation, the experts asked to add an important “teaching goal” indicator to the teacher questionnaire, and eight secondary “teaching goals” indicators: “The Benefits of Learning Mental Health Network,” “The Concept of Learning Mental Health Network,” “Training Objectives of Mental Health Education Network,” “Online Self-Help and Collaboration,” “Online Self-Help Concept,” and Communication and Cooperation.” At the same time, eight secondary indicators of “online time period,” “online emotional motivation,” “online emotional experience,” “online browsing content,” “satisfaction with online mental health education,” “online self-help and mutual assistance,” “online self-help and mutual assistance content,” and “impact of nonmainstream culture” were added to the college students' questionnaire. In addition, the “network mental health education content” is divided into three secondary indicators: “network mental health education curriculum content,” “online measurement and evaluation content,” and “online psychological counseling content,” and the experts have modified its option setting.

In the second round of formal consultation, the secondary indicator of “impact of nonmainstream culture” was deleted according to the deletion standard. After three rounds of expert consultation, the educators' questionnaire selected six first-class indicators of “feasibility,” “management system,” “support system,” “education objective system,” “education system,” and “education effect evaluation,” and the following 30 second-class indicators. The questionnaire of college students selected four first-class indicators of “network use,” “use intention and demand,” “use status and effect,” and “construction of education system,” and the following 32 second-class indicators.

#### 3.4.2. Index Weight

The weight scores of the indicators given by experts were normalized. The calculation shows that the weights of the six primary indicators in the educator questionnaire are close to each other. Among them, “feasibility,” “support system,” and “education system” have the highest weight of 0.1800 and “management system” has the lowest weight of 0.1400. Among the secondary indicators, the top three items with the highest weight are “training objectives of online mental health education,” “effectiveness of online mental health education,” and “values of online mental health education,” and those with the lowest weight are “online self-help and mutual assistance content,” “online measurement and evaluation content,” and “online psychological counseling content.” In the teacher questionnaire, the weights of the two concepts of “Internet use” and “rules and regulations” are 0.2625, and the weights of the concepts of “Internet use,” “use goals and needs,” and “educational development” are 0.2375. On the second scale, the top five most important criteria were “terms used in online mental health education,” “significantly affecting the use of online mental health education,” ” the importance of online mental health education,” “need for online mental health education,” and “interest in doing online mental health education.” The most important are “online self-help and content sharing services,” “online mental health counseling content,” and “online content measurement” (see Tables 5 and 6 for details).

Based on literature research and case interviews, combined with the data obtained from expert consultation, and according to the selection principles of suitability, systematicness, feasibility, and effectiveness indicators, a questionnaire on mental health education for college students in a city (educators/college students) is compiled. In the questionnaire for educators, the five-grade scoring system is adopted for the four secondary indicators of importance, need, and willingness to carry out and effect perception, and the multichoice method is adopted for the four secondary indicators of appropriate contents of online courses, online measurement and evaluation, online psychological counseling, and online self-help and mutual assistance. The questionnaire for college students includes three parts: demographic characteristics, Internet use, and Internet mental health education. Among them, the five-level scoring system is adopted for the seven secondary indicators of importance, need, understanding, willingness to use, frequency of use, satisfaction, and effect perception, and the multichoice method is adopted for the four secondary indicators of online courses, online measurement and evaluation, online psychological counseling, and online self-help and mutual assistance. At the same time, an open question was set at the end of the two types of questionnaires to collect the suggestions of educators and college students on online mental health education.

## 4. Result Analysis

Nine experts were invited to distribute the electronic questionnaire through the questionnaire star in multiple colleges. The quality of questionnaire filling is controlled by means of question type design, option setting, IP control, filling logic, screening rules, and so on. A total of 932 questionnaires were collected from college students in this study, and 23 questionnaires with a duration of less than 180 seconds were excluded. A total of 909 valid questionnaires were compiled, with an effective rate of 97.53%; at the same time, a total of 34 teachers were asked questions, excluding 0 questionnaires with a duration of less than 120 seconds, a total of 34 active questionnaires, with 100% quality assurance.

Among the surveyed college students, 561 (61.72%) were women and 348 (38.28%) were men. Their majors covered liberal arts, science, engineering, agriculture, economics, management, medicine, art, and other disciplines. The grades were widely distributed, mainly freshmen (37.29%) and sophomores (30.03%). The proportion of non-only-children (75.91%) was high, and the proportions of urban and rural students were basically the same (see Tables 7–11 for details).

Cronbach's Alpha coefficient is an internal belief commonly used to measure the consistency of a questionnaire. It is generally believed that if the coefficient is greater than 0.7, the reliability of the questionnaire is high, and if the coefficient is greater than 0.8, the reliability of the questionnaire is very good [19].

### 4.1. Reliability Test of Educators' Questionnaire

SPSS 170 analysis results show that [11,20] total Cronbach's Alpha coefficient of teacher query is greater than 0.8, and Cronbach's Alpha coefficient of query length is 0.7, indicating that the questionnaire is based on research (see Figure 2 for details) [21].

### 4.2. Reliability Test of College Student Questionnaire

Overall Cronbach's Alpha coefficient of the college students' questionnaire was 0.845, and Cronbach's Alpha coefficients of the four major questionnaires were all greater than 0.7. As can be seen, the questionnaire is research-based (see Figure 3 for details) [22].

Validity reflects the consistency between the test results and the tester's real behavior. The higher the validity is, the more accurate and effective the test can be. This research questionnaire is formulated through expert consultation, and experts mainly evaluate it with professional knowledge. It can be considered to have good valid content. Meanwhile, state analysis was used to evaluate the feasibility of the questionnaire. First, by KMO and Bartlett's test of sphericity, when the KMO data is greater than 0.7, it indicates that the questionnaire is suitable for analysis [23].

The KMO test measures different data in terms of correlation coefficients and semicorrelation coefficients. When the sum of squares of the simple correlation coefficients of all variables is equal to the number of squares of the fractional correlation coefficients, the stronger the correlation of variables is, the more suitable it is for principal component analysis. Otherwise, it is not suitable for critical analysis.

Let (*X*_*i*_, *Y*_*i*_)(*i*=1,2,…, *n*) be the sample taken from the population; the calculation formula of Pearson simple linear correlation coefficient of the sample is as follows [24]:

(2) $$\begin{array}{c} \rho =\frac{\sum_{i=1}^{n}\left(X_{i}-\bar{X}\right)\left(Y_{i}-\bar{Y}\right)}{\sqrt{\sum_{i=1}^{n}{\left(X_{i}-\bar{X}\right)}^{2}}\sqrt{\sum_{i=1}^{n}{\left(Y_{i}-\bar{Y}\right)}^{2}}}, \end{array}$$

(3) $$\begin{array}{c} \bar{X}=\frac{1}{n}\sum_{i=1}^{n}X_{i}, \end{array}$$

(4) $$\begin{array}{c} \bar{Y}=\frac{1}{n}\sum_{i=1}^{n}Y_{i}. \end{array}$$

The partial correlation coefficient is calculated by the correlation coefficient of two variables in fixing the strength of the other variable, and it can affect the degree of linear correlation of one of the two variables under the influence of the other fixed differently. The formula for the partial correlation coefficient is as follows:

(5) $$\begin{array}{c} r_{xy,z_{1}}=\frac{r_{xy}-r_{xz_{1}}r_{yz_{1}}}{\sqrt{\left(1-r_{xz_{1}}^{2}\right)\left(1-r_{yz_{1}}^{2}\right)}}, \end{array}$$

(6) $$\begin{array}{c} \frac{r_{xy}-r_{xz_{1}}r_{yz_{1}}}{\sqrt{\left(1-r_{xz_{1}}^{2}\right)\left(1-r_{yz_{1}}^{2}\right)}}=h=1, \end{array}$$

(7) $$\begin{array}{c} r_{xy,z_{1}z_{2}z_{3}\ldots z_{h}}=\frac{r_{xy,z_{1}z_{2}z_{3}\ldots z_{h-1}}-r_{xz_{h},z_{1}z_{2}z_{3}\ldots z_{h-1}}r_{yz_{h},z_{1}z_{2}z_{3}\ldots z_{h-1}}}{\sqrt{\left(1-r_{xz_{h},z_{1}z_{2}z_{3}\ldots z_{h-1}}^{2}\right)\left(1-r_{yz_{h},z_{1}z_{2}z_{3}\ldots z_{h-1}}^{2}\right)}}, \end{array}$$

(8) $$\begin{array}{c} r_{xy,z_{1}z_{2}z_{3}\ldots z_{h}}=h\geq 2, \end{array}$$

where *r*_(*xy*,*z*_1_)_ is the number of stable exchanges; *r*_(*xy*, *z*_1_*z*_2_*z*_3_ … *z*_*h*_)_ is the fixed exchange; and *r*_(*xy*, *z*_1_*z*_2_*z*_3_ … *z*_*h*_)_ is the simple correlation coefficient of the variable.

Assuming that the squared equation of the average correlation coefficient is P and the squared equation of the average correlation coefficient is *r*, the standard calculation of the KMO test statistic is

(9) $$\begin{array}{c} M=\frac{P}{P+R}. \end{array}$$

The Bartlett sphericity test starts with the relative coefficient matrix of the original matrix, and its null hypothesis is that the relative coefficient matrix is the identity matrix. The statistics for Bartlett's test of sphericity are determined based on the coefficient matrix. The standard calculation of statistics is as follows [25]:

(10) $$\begin{array}{c} \emptyset =\det\left(\text{O}\right), \end{array}$$

(11) $$\begin{array}{c} \emptyset =\left\lfloor \text{O}\right\rfloor . \end{array}$$

According to the observed values of degrees of freedom and statistics, the corresponding concomitant probability can be approximately obtained by querying the chi square distribution table.

### 4.3. Validity Test of Educators' Questionnaire

As shown in Table 12, the KMO test score of the teacher questionnaire was 0.722, the Bartlett sphericity test value was 590.794, and the *p* value was 0.000 (*P* < 0.01), indicating that the questionnaire was suitable for analysis.

### 4.4. Validity Test of College Student Questionnaire

As shown in Table 13, the test score of KMO's test students is 0.798, the score of Bartlett's spherical test is 1298.768, and the *p* value is 0.000 (*P* < 0.01), indicating that a questionnaire is needed for identification.

As shown in Tables 14–16, 44.12% of educators believe that the values with the educated as the main body should be established, and 32.35% believe that the values with the society as the main body should be established. Most educators believe that they should adhere to the educational concept of all-round development (41.18%) and people-oriented (26.47%). The training objectives are to improve college students' mental health quality (41.18%), popularize mental health knowledge (23.53%), identify and find mental problems (23.53%), and prevent and reduce mental crisis (11.76%).

## 5. Conclusion

Through the investigation and data analysis of educators and college students, the following conclusions are drawn:

1. Surfing the Internet has become a daily habit of college students. The behavior of using the Internet is more rational. They pursue entertainment, relaxation, and access to information. The mindset is simple and pleasant, and the mindset is further influenced by college students' interest in using online psychosocial education.
2. Educators and college students have strong needs and willingness for online mental health education, while the low security significantly affects the needs of both sides. Although most college students have received online mental health education, their understanding, satisfaction, and effectiveness of online mental health education are still low, and there is still a large demand gap.
3. On the basis that the needs of educators and college students are basically the same, there are also some differences. In terms of content, the needs of educators and college students are highly overlapped in self-awareness, professional psychology and career planning, interpersonal relationship, and social support. In terms of form, they all think that video and pictures are the main means. In the choice of educational channels, educators tend to prefer campus websites, while college students tend to prefer social software.
4. In the construction of mental education in online education, educators believe that it is necessary to increase hardware products, network environment, funds, and office funds, serve as the chairman of the school party committee, the Ministry of Education, and the Ministry of Students, and have one intellectual team with mental health background.

From the perspective of the thesis and the benefits of online education, this article proposes a series of advocacy efforts aimed at improving student mental health education and promoting online learning efforts.

## Figures and Tables

**Figure 1:** Technical roadmap.

**Figure 2:** Reliability test (educator questionnaire).

**Figure 3:** Reliability test (college student questionnaire).

**Table 1:** Basic information of consulting experts.

Basic information		Number of people	Proportion (%)
Gender	Male	2	22.22
	Female	7	77.78

Age	30–39 years old	3	33.33
	40–49 years old	1	11.11
	50–59 years old	4	44.44
	Over 60 years old	2	22.22

Major	Psychology	6	66.67
	Management	1	11.11
	Education	1	11.11
	Medical science	1	11.11

Education	Undergraduate	1	11.11
	Master's degree	4	44.44
	Doctoral candidate	4	44.44

Occupation	Teacher	8	88.89
	Psychological consultation teacher	1	11.11

Title	Intermediate	2	22.22
	Deputy senior	5	55.56
	Positive advanced	2	22.22

Years of service	5–10 years	3	33.33
	11–15 years	2	22.22
	16–20 years	1	11.11
	More than 20 years	3	33.33

**Table 2:** Quantitative value of expert authority coefficient.

Familiarity	Quantization coefficient (Cs)	Judgment basis	Quantization coefficient (Ca)		
			Large	Middle	Small
Very familiar	1.0	Theoretical basis	0.3	0.2	0.1
Quite familiar	0.8	Practical basis	0.5	0.4	0.3
Commonly	0.6	Peer understanding	0.1	0.1	0.05
Less familiar	0.4	Intuitive judgment	0.1	0.1	0.05
Unfamiliar	0.2				

**Table 3:** Coordination coefficient of expert opinions (questionnaire for educators).

Index	Scoring item	N	The second round of formal consultation			The third round of formal consultation		
			*W*	*X* ^*2*^	*p*	*W*	*X* ^*2*^	*p*
Primary index	Necessity	6	0.601	27.091	0.000	0.653	19.591	0.000
	Feasibility	6	0.488	22.006	0.000	0.626	18.780	0.000
Secondary index	Necessity	30	0.418	112.860	0.000	0.844	151.742	0.006
	Feasibility	30	0.383	103.410	0.000	0.836	150.300	0.021
Tertiary indicators	Necessity	36	0.433	139.967	0.000	0.720	155.304	0.000
	Feasibility	36	0.418	135.108	0.000	0.707	152.713	0.000

**Table 4:** Coordination coefficient of expert opinions (questionnaire for college students).

Index	Scoring item	N	The second round of formal consultation			The third round of formal consultation		
			W	X^2^	P	W	X^2^	P
Primary index	Necessity	4	0.787	21.249	0.001	0.853	23.031	0.000
	Feasibility	4	0.699	18.845	0.000	0.753	20.304	0.006

Secondary index	Necessity	33	0.440	130.978	0.000	0.615	176.832	0.000
	Feasibility	33	0.387	114.939	0.000	0.603	173.375	0.000

Tertiary indicators	Necessity	37	0.585	194.472	0.001	0.738	239.436	0.000
	Feasibility	37	0.517	172.160	0.000	0.705	228.421	0.000

**Table 5:** Index weight (educator questionnaire).

Primary index	Weight coefficient	Secondary index	Weight coefficient
Feasibility index	0.18	The importance of learning about mental networks	0.0413
		The degree of need for psychiatric network education	0.0413
		Interest in online mental health education	0.0308
		Factors of attracting network mental health education	0.0324
		Factors affecting the development of network mental health education	0.0342
Management system indicators	0.14	System construction	0.0518
		Organizational leadership	0.0490
		Supervision	0.0392
Support system indicators	0.18	Teaching staff	0.0450
		Supervision system	0.0396
		Financial support	0.0414
		Working conditions	0.0288
		Network presentation level	0.0252
Education objective system indicators	0.16	Values of network mental health education	0.0544
		Concept of network mental health education	0.0480
		Training objectives of network mental health education	0.0576
Education system indicators	0.18	Suitable channels for network mental health education	0.0166
		Activity-appropriate online mental health education	0.0176
		Essential information for the mental health education network	0.0176
		Network mental health education course	0.0176
		Suitable content of network mental health education course	0.0155
		Online measurement and evaluation	0.0151
		Suitable content for online measurement and evaluation	0.0112
		Online psychological counseling	0.0166
		Suitable content of online psychological counseling	0.0119
		Online self-help and mutual assistance	0.0130
		Suitable content for online self-help and mutual assistance	0.0097
Evaluation index of educational effect	0.16	Effectiveness of network mental health education	0.0557
		Factors affecting the effect of network mental health education	0.0522
		Evaluation method of network mental health education effect	0.0522
Feasibility index	0.18	Importance of network mental health education	0.0413
		The degree of need for network mental health education	0.0413
		Willingness to carry out online mental health education	0.0308
		Factors of attracting network mental health education	0.0324
		Factors affecting the development of network mental health education	0.0342
Management system indicators	0.14	System construction	0.0518
		Organizational leadership	0.0490
		Supervision	0.0392
Support system indicators	0.18	Teaching staff	0.0450
		Supervision system	0.0396
		Financial support	0.0414
		Working conditions	0.0288
		Network presentation level	0.0252
Education objective system indicators	0.16	Values of network mental health education	0.0544
		Concept of network mental health education	0.0480
		Training objectives of network mental health education	0.0576
Education system indicators	0.18	Suitable channels for network mental health education	0.0166
		Network mental health education is suitable for carrying out activities	0.0176
		Suitable forms of network mental health education	0.0176
		Network mental health education course	0.0176
		Suitable content of network mental health education course	0.0155
		Online measurement and evaluation	0.0151
		Suitable content for online measurement and evaluation	0.0112
		Online psychological counseling	0.0166
		Suitable content of online psychological counseling	0.0119
		Online self-help and mutual assistance	0.0130
		Suitable content for online self-help and mutual assistance	0.0097
Evaluation index of educational effect	0.16	The effectiveness of psychological network education	0.0557
		The importance of learning the benefits of the mental health network	0.0522
		Psychoeducational network evaluation	0.0522

**Table 6:** Index weight (college student questionnaire).

Primary index	Weight coefficient	Secondary index	Weight coefficient
Network usage indicators	0.2625	Internet access equipment	0.0230
		Internet frequency	0.0315
		Average online time per day	0.0381
		Internet habit time period	0.0282
		Main purpose of surfing the Internet	0.0308
		Online emotional motivation	0.0249
		Online emotional experience	0.0249
		Engaging in activities online	0.0289
		Browsing content online	0.0322
Use intention and demand indicators	0.2375	The importance of learning about mental networks	0.0455
		The degree of need for network mental health education	0.0475
		Willingness to carry out online mental health education	0.0475
		The main attraction of studying mental networks	0.0505
		Important factors affecting the development of mental health education network	0.0475
Application status and effect indicators	0.2625	Understanding network mental health education	0.0348
		Frequent use of online mental health education	0.0420
		Most people use online mental health information	0.0354
		The effectiveness of psychological network education	0.0348
		Satisfaction degree of network mental health education	0.0420
		Factors affecting the effect of network health education	0.0354
		Psychoeducational network evaluation	0.0381
Educational system construction indicators	0.2375	Suitable channels for network mental health education	0.0214
		Network mental health education is suitable for carrying out activities	0.0232
		Essential information for the mental health education network	0.0232
		Mental health network	0.0232
		Suitable content of network mental health education course	0.0196
		Online measurement and evaluation	0.0220
		Suitable content for online measurement and evaluation	0.0154
		Online psychological counseling	0.0214
		Suitable content of online psychological counseling	0.0137
		Online self-help and mutual assistance	0.0184
		Suitable content for online self-help and mutual assistance	0.0131
Network usage indicators	0.2625	Internet access equipment	0.0230
		Internet frequency	0.0315
		Average online time per day	0.0381
		Internet habit time period	0.0282
		Main purpose of surfing the Internet	0.0308
		Online emotional motivation	0.0249
		Online emotional experience	0.0249
		Engaging in activities online	0.0289
		Browsing content online	0.0322
Use intention and demand indicators	0.2375	Importance of network mental health education	0.0455
		The degree of need for network mental health education	0.0475
		Willingness to carry out online mental health education	0.0475
		Factors of attracting network mental health education	0.0505
		Factors affecting the development of network mental health education	0.0475
Application status and effect indicators	0.2625	Understanding network mental health education	0.0348
		Frequency of using network mental health education	0.0420
		Most used online mental health education activities	0.0354
		Effectiveness of network mental health education	0.0348
		Satisfaction degree of network mental health education	0.0420
		Factors affecting the effect of network health education	0.0354
		Evaluation method of network mental health education effect	0.0381
Educational system construction indicators	0.2375	Suitable channels for network mental health education	0.0214
		Network mental health education is suitable for carrying out activities	0.0232
		Suitable forms of network mental health education	0.0232
		Network mental health education course	0.0232
		Suitable content of network mental health education course	0.0196
		Online measurement and evaluation	0.0220
		Suitable content for online measurement and evaluation	0.0154
		Online psychological counseling	0.0214
		Suitable content of online psychological counseling	0.0137
		Online self-help and mutual assistance	0.0184
		Suitable content for online self-help and mutual assistance	0.0131

**Table 7:** Demographic characteristics of survey samples (gender).

Gender	Number of people	Proportion (%)
Male	348	38.28
Female	561	61.72

**Table 8:** Demographic characteristics of survey samples (major).

Major	Number of people	Proportion (%)
Engineering	219	24.09
Management	171	18.81
Neo-Confucianism	165	18.15
Literature	87	9.57
Economics	84	9.24
Agronomy	54	5.94
Law	39	4.29
Art studies	33	3.63
Medical science	33	3.63
Education	15	1.65
Philosophy	9	0.99

**Table 9:** Demographic characteristics of survey samples (grade).

Grade	Number of people	Proportion (%)
First year	339	37.29
Second year	273	30.03
Third year	171	18.81
Fourth year	90	9.90
Fifth year	36	3.96

**Table 10:** Demographic characteristics of survey samples (only-child).

Only-child	Number of people	Proportion (%)
Yes	219	24.09
No	690	75.91

**Table 11:** Demographic characteristics of survey samples (place of origin).

Place of origin	Number of people	Proportion (%)
Countryside	483	53.14
City	426	46.86

**Table 12:** KMO and Bartlett's test (educator questionnaire).

Kaiser–Meyer–Olkin measurement of flow velocity		0.722
Bartlett's sphericity test	Approximate chi square	590.794
	df	300
	*P*	0.000

**Table 13:** KMO and Bartlett's test (college student questionnaire).

Kaiser–Meyer–Olkin measure of sampling adequacy		0.798
Bartlett's sphericity test	Approximate chi square	1298.768
	Df	351
	P	0.000

**Table 14:** Education objective system (educational values).

Education objective system indicators	Number of people	Proportion (%)
Values with the educated as the main body	15	44.12
Values with educators as the main body	4	11.76
School-centered values	4	11.76
Values with society as the main body	11	32.35

**Table 15:** Education objective system (education concept).

Education objective system indicators	Number of people	Proportion (%)
People-oriented concept	14	41.18
Comprehensive development concept	9	26.47
Concept of quality education	6	17.65
Personalized concept	3	8.82
Open concept	2	5.88

**Table 16:** Education objective system (training objective).

Education objective system indicators	Number of people	Proportion (%)
Popularizing mental health knowledge	8	23.53
Improving college students' mental health quality	14	41.18
Identifying and finding psychological problems	8	23.53
Prevention and reduction of psychological crisis	4	11.76

## Data Availability

The labeled dataset used to support the findings of this study is available from the author upon request.

## References

[1] Wang Z., Yu N. (2021). Education data-driven online course optimization mechanism for college student. *Mobile Information Systems*.

[2] Ding Y., Chen X., Fu Q., Zhong S. (2020). A depression recognition method for college students using deep integrated support vector algorithm. *IEEE Access*.

[3] Bedi P., Gole P., Dhiman S., Gupta N. (2020). Smart contract based central sector scheme of scholarship for college and university students. *Procedia Computer Science*.

[4] Awalya A., Suharso S., Nugraha Y. P., Kunwijaya I., Syifa L. (2020). The identification of postgraduate students mental health in terms of gender, age, and education level. *Solid State Technology*.

[5] Gong K. (2020). Extensible strategies and their performance for mental health education in colleges. *International Journal of Emerging Technologies in Learning (iJET)*.

[6] Taghvaei N., Masoumi B., Keyvanpour M. R. (2021). Analytical framework for mental health feature extraction methods in social networks. *Intelligent Decision Technologies*.

[7] Zhang J. (2021). A study on mental health assessments of college students based on triangular fuzzy function and entropy weight method. *Mathematical Problems in Engineering*.

[8] Zhao Y., Tang Q. (2021). Analysis of influencing factors of social mental health based on big data. *Mobile Information Systems*.

[9] Allen S. (2021). Probing the future of psychedelics for mental health. *IEEE Pulse*.

[10] Alégroth E., Gorschek T., Petersen K., Mattsson M. (2020). Characteristics that affect preference of decision models for asset selection: an industrial questionnaire survey. *Software Quality Journal*.

[11] Marcial D. E., Launer M. A. (2021). Test-retest reliability and internal consistency of the survey questionnaire on digital trust in the workplace. *Solid State Technology*.

[12] Pereira C., Sachidananda H. K. (2022). Impact of industry 4.0 technologies on lean manufacturing and organizational performance in an organization. *International Journal on Interactive Design and Manufacturing*.

[13] Yasui A., Numada M. (2021). A report of the questionnaire survey on awareness of covid-19 and shelters. *Journal of Disaster Research*.

[14] Yusuwan N. M., Adnan H., Rashid Z. Z. A., Ismail W. N. W., Mahat N. A. A. (2021). Towards a successful extension of time (eot) claim: a consensus view of construction professionals via a modified delphi method. *Engineering Journal*.

[15] Khalilzadeh M., Shakeri H., Zohrehvandi S. (2021). Risk identification and assessment with the fuzzy dematel-anp method in oil and gas projects under uncertainty. *Procedia Computer Science*.

[16] Amirghodsi S., Naeini A. B., Makui A. (2020). An integrated delphi-dematel-electre method on gray numbers to rank technology providers. *IEEE Transactions on Engineering Management*.

[17] Li H., Li B., Yang G., Chen C., Chen Y., Zhao C. (2020). Evaluating the regulatory environment of overseas electric power market based on a hybrid evaluation model. *International Journal of Fuzzy Systems*.

[18] Crispim D. L., Progênio M. F., Fernandes L. L. (2022). Proposal for a tool for assessing access to water in rural communities: a case study in the brazilian semi-arid. *Environmental Management*.

[19] Jing B. (2022). Comparative study on the validity of monitoring test indexes of healthy fitness cardiopulmonary track and field sensor. *EURASIP Journal on Applied Signal Processing*.

[20] Olorunda S. (2020). Security education for sustainable development and peaceful coexistence in southwest Nigeria. *Journal of Management Information Systems*.

[21] Swamynathan K., Singadurai A., Sivakumar P. (2021). Sterilization of dry-type transformer winding by conducting short-circuit test in nuclear power plant: a case study. *Journal of the Institution of Engineers: Serie Bibliographique*.

[22] Ebi A., Reisolu L. (2022). Adaptation of self-assessment instrument for educators’ digital competence into turkish culture: a study on reliability and validity. *Technology, Knowledge and Learning*.

[23] Rubia M., Rus-Casas C., Bueno-Rodriguez S., Aguilar-Pena J. D., Eliche-Quesada D. (2021). Study of the entrepreneurial attitudes of stem students. *IEEE Access*.

[24] Chen C., Wang G., Guan H., Liang Y.-C., Tellambura C. (2020). Transceiver design and signal detection in backscatter communication systems with multiple-antenna tags. *IEEE Transactions on Wireless Communications*.

[25] Magalhes T. M., Gallardo D. (2020). Bartlett and bartlett-type corrections for censored data from a weibull distribution. *Statistics and Operations Research Transactions*.

